The article "Influence of Sevoflurane Inhalation Anesthesia on Clinical Outcomes of Morbidly Obese Patients Undergoing Laparoscopic Bariatric Surgery" was published in 2022. Journal: Evid Based Complement Alternat Med.

# Influence of Sevoflurane Inhalation Anesthesia on Clinical Outcomes of Morbidly Obese Patients Undergoing Laparoscopic Bariatric Surgery

**DOI:** 10.1155/2022/1408948

**Published:** 2022-09-06

**Authors:** Wei Li, Ying Zhang, Jianrui Lv, Yong Zhang, Jie Bai

**Affiliations:** Department of Anesthesia, The Second Affiliated Hospital of Xi'an Jiaotong University, Xi'an 710004, Shaanxi, China

## Abstract

**Background:**

Morbid obesity is one of the fastest-growing subgroups of obesity and is associated with high mortality, with an estimated 2.8 million people dying from obesity each year.

**Objective:**

This research sets out to elucidate the impact of sevoflurane (Sevo) inhalation anesthesia on the clinical outcome of morbidly obese (MO) patients undergoing laparoscopic bariatric surgery (LBS).

**Methods:**

A retrospective study was conducted on 150 MO patients undergoing LBS in the Second Affiliated Hospital of Xi'an Jiaotong University from November 2019 to November 2021. According to the difference of anesthesia methods, 100 patients with Sevo anesthesia were set as group A, and 50 patients with propofol (P) anesthesia were set as group B. Intergroup comparisons were performed in terms of eye-opening time, tracheal intubation removal time, directional force recovery, heart rate (HR), mean arterial pressure (MAP), peak airway pressure (P_peak_), plateau pressure (P_plat_), standard time out of PACU, postoperative food intake (FI), length of stay (LOS), and complication rate.

**Results:**

Group A had a shorter time to open eyes, remove tracheal intubation, and restore directional force than Group B, with better recovery of HR, MAP, P_peak_, and P_plat_. Group A was also superior to Group B in the standard time out of PACU, postoperative FI, and LOS, with a lower complication rate.

**Conclusions:**

Sevo inhalation anesthesia is more effective and safer for MO patients undergoing LBS.

## 1. Introduction

Obesity is a chronic condition defined as body mass index (BMI) > 30 kg/m^2^, of which morbid obesity, defined as body mass index (BMI) > 40 kg/m^2^, is one of the fastest-growing subgroups [1, 2]. In recent years, there has been a gradual increase in the rate of obesity, accompanied by a dramatic increase in obesity-related metabolic diseases, including type 2 diabetes [3, 4], and ileal Crohn's disease [5]. Morbid-obesity-related conditions such as stroke, acute myocardial infarction, hypertension, type 2 diabetes, hyperlipidemia, and obstructive sleep apnea are associated with high mortality rates, with approximately 2.8 million deaths per year among obesity-affected adults [6, 7]. In recent years, treatments for morbid obesity, such as weight-reducing drugs and insulin resistance therapy, have been constantly improved. But bariatric surgery is still very important for morbidly obese (OB) patients. Therefore, this study aims to improve the surgical protocol for MO patients in order to provide a better choice for the clinical treatment of such a patient population.

Bariatric surgery has long been considered the most effective method to treat severe obesity and its complications, with mortality rates falling below 0.1 per cent in the past decade [8]. Currently, the number of patients undergoing bariatric surgery is steadily increasing globally due to increased demand, accessibility, and advances in laparoscopic surgery. However, laparoscopic surgery is associated with a high incidence of complications that can predispose patients to readmission or even death in the absence of strict protection measures [9]. It is shown that appropriate anesthesia can speed up patient recovery and reduce the risk of infection [10]. Therefore, anesthesia for patients is very important. Among them, the application of sevoflurane (Sevo) inhalation anesthesia is becoming more and more extensive [11]. However, a randomized controlled study suggested that Sevo may produce stress responses of varying degrees during laparoscopic surgery [12]. And among previous studies on Sevo's application in laparoscopic surgery, there are relatively few studies investigating its role in MO patients. Accordingly, in this study, we combined a series of indicators to study the impact of this anesthesia approach on the clinical outcomes of laparoscopic bariatric surgery (LBS) for MO patients.

## 2. Methods

### 2.1. General Data

From November, 2019 to November, 2021, 150 MO patients undergoing LBS were selected and assigned to Sevo anesthesia Group A (*n* = 100) and Propofol (P) anesthesia Group B (*n* = 50) according to the difference in inhaled anesthetics during surgery. Inclusion criteria: the participants were all MO patients undergoing LBS in our hospital, with BMI >40 kg/m^2^, normal psychology, and communication ability, as well as the consent and signed relevant agreements from patients and their families. Exclusion criteria: surgical contraindications; drug allergies or endocrine system diseases; history of cerebral hemorrhage and cerebral infarction within 1 year; and severe heart and brain organ lesions. This research was conducted after obtaining approval from the Ethics Committee of the Second Affiliated Hospital of Xi'an Jiaotong University.

### 2.2. Methods

All patients were fasted for 10h and abstained from drinking for 6h preoperatively. The airway was established by tracheal intubation before anesthesia, and preoperative airway pressure monitoring and results recording were performed. All patients underwent LBS in the supine position. Pneumoperitoneum was established during the operation, and pulmonary recruitment maneuver (PRM) were performed every 30 min. The steps of PRM are as follows: (1) The respiration rate and pressure limit were set as 8 beats/min and 40 cm H_2_O, respectively; (2) The positive end-expiratory pressure (PEEP) was set as 5 cm H_2_O when initiating the ventilation, which was increased by 10 cm H_2_O and 15 cm H_2_O after 5 times of ventilation to gradually increase the tidal volume (TV) until the peak airway pressure (P_peak_) reached 40 cm H_2_O; (3) TV was restored to the level before PRM by gradually reducing the PEEP to 10 cm H_2_O, 5 cm H_2_O and 0 cm H_2_O. Scopolamine was injected intramuscularly 30 min before anesthesia. After opening the patient's venous access, 10 ml/(kg·h) Sodium Lactate Ringer's Injection was administered intravenously, and the mask oxygen inhalation was maintained at 2–4 L/min. The patient's heart rate (HR) and mean arterial pressure (MAP) were detected by puncture and catheterization around the left artery under local anesthesia. Besides, the patient was given an iv bolus of 0.2 mg/kg atracurium and 0.4 g/kg sufentanil. Furthermore, Group B was given 3 mg/kg P, while Group A was given Sevo with an initial and a maximum inhalation concentration of 7.0% and 8.0%, respectively. The patient underwent mechanical ventilation after spontaneous breathing disappeared, with a respiratory ratio of 1 : 1.5, a frequency of 12 times/min and a TV of 8–9 ml/kg. The anesthesia concentration was adjusted according to the bispectral index scale (BIS), HR, and blood pressure (BP) of patients, and BIS was maintained at 40–50 to keep the HR stable. Urapidil was given if BIS <40 and BP was 120% above normal. Phenylephrine was administered if the patient's BP was below 70% of normal; in cases with HR > 90 beats/min, esmolol was given, while atropine was given to those with HR < 50 beats/min. The anesthetic concentration was increased once BIS >50 was observed; 5 *μ*g of sufentanil was administered when the patient's HR was more than 90 beats/min or the BP was 120% higher than normal. Phenylephrine was given if BP was below 70% of normal. And in those with a HR < 50 beats/min, atropine was given. The inhalation of P and Sevo was gradually reduced 15 min before surgery, and withdrawn after the completion of the operation. When patients resumed spontaneous breathing, 0.5 mg atropine, and 1 mg neostigmine were injected. Airway pressures were remonitored in all patients postoperatively and the results were recorded.

### 2.3. Endpoints

#### 2.3.1. Anesthesia Recovery Time

The times of eye-opening time (from stopping anesthetics to being awakened to open eyes), the time of tracheal intubation removal (from withdrawal of anesthetics to removal of bronchial intubation) and the time of restoring orientation (from withdrawal of anesthetics to blinking and coughing as instructed) were observed and recorded.

#### 2.3.2. Hemodynamics

The preoperative and postoperative hemodynamics (HR, MAP) were compared.

#### 2.3.3. Pulmonary Function (PF)

The pre- and posttreatment PF (P_peak_, plateau pressure (P_plat_)) of the two groups was compared.

#### 2.3.4. Postoperative Recovery

The two cohorts were also compared in terms of postoperative recovery as assessed by the following indices: the standard time out of postanesthesia care unit (PACU), postoperative food intake, and length of stay (LOS).

#### 2.3.5. Complication Rate

The postoperative complications were compared. The related indicators included nausea, vomiting, labored breathing, and chills.

### 2.4. Statistical Processing

SPSS19.0 (Asia Analytics Formerly SPSS China) and GraphPad Prism 6 (GraphPad Software, San Diego, USA) were employed for comprehensive statistical analysis and visualization of data, respectively. Enumeration data (sex, family status, etc.), denoted by number of cases/percentage (n/%), were compared by the *χ*2 test; the *t*-test was used to identify the difference of quantitative data (age, BMI, etc.) denoted by ($\bar{x}$± *s*). A significance level of *P* < 0.05 was used in this study.

## 3. Results

### 3.1. General Information

Groups A and B differed insignificantly in a series of general data like sex, age, BMI, family status, and drinking (yes/no) (*P* > 0.05) (Table 1).

### 3.2. Recovery Time from Anesthesia

After comparing patients' anesthesia recovery, it was found that the eye-opening time, tracheal intubation removal time and directional force recovery time were significantly shorter in Group A compared with Group B, with statistical significance (*P* < 0.05) (Figure 1).

### 3.3. Hemodynamics

The comparison of patients' hemodynamics revealed statistically higher posttreatment HR and MAP in Group A versus Group B, showing statistical significance (*P* < 0.05) (Figure 2).

### 3.4. PF

The intergroup comparison of patients' PF also determined statistically lower posttreatment P_peak_ and P_plat_ in Group A compared with Group B (*P* < 0.05) (Figure 3).

### 3.5. Comparison of Postoperative Recovery

The comparison of postoperative recovery between groups showed statistically shorter standard time out of PACU, postoperative eating time and LOS in Group A compared with Group B (*P* < 0.05) (Figure 4).

### 3.6. Complication Rate

Comparing the complication rate between Groups A and B, we found a statistically lower postoperative complication rate in Group A (*P* < 0.05) (Table 2).

## 4. Discussion

Morbid obesity is an extremely challenging disease that affects every aspect of patients' lives [13]. Minimally invasive bariatric surgery is becoming increasingly popular because of the disappointing long-term outcomes of medical and behavioral interventions [14]. Of these, LBS is by far the most popular, accounting for more than 50 to 60 percent of global bariatric surgery [15]. Although various clinical studies have shown that LBS has a favorable effect on weight reduction, it will still bring a series of complications if not performed with good anesthesia [16, 17]. In this section, we will discuss the anesthetic effect of Sevo based on the findings of this clinical study.

From the perspective of anesthesia recovery time, Group A using Sevo had shorter eye-opening time, earlier tracheal intubation removal, and faster directional force recovery than Group B using *P*. Although anesthesia benefits various surgical procedures and patients, improper anesthesia puts patients at greater risk of neurocognitive impairment and even reduces their processing speed and impairs their fine motor abilities [18]. In an animal model, neuroinflammation and other damage in addition to cognitive impairment, have been found if anesthetics are poorly chosen [19, 20]. So, the choice of anesthetics is very important in surgery. Sevo, a recognized inhalation anesthetic extensively used in various surgical procedures [21], has antioxidant stress and anti-inflammatory properties, which are important in protecting organs from stress-induced damage [22]. *P*, another drug most commonly used in international anesthesia and intensive care, also has good pharmacokinetics and rapid and reversible sedation [23]. However, it comes with obvious disadvantages, as it will not only cause complications such as severe metabolic acidosis and bradycardia-induced cardiac arrest, but even lead to rhabdomyolysis and acute kidney injury (AKI), all of which compromise the anesthetic effect [24]. Therefore, the recovery from anesthesia was faster in Group A. And combining the results of PF and hemodynamics, it is clear that Sevo used in Group A protected the lungs and heart from pressure, resulting in better PF and hemodynamics than Group B. It suggests that not only may the effects of anesthesia be impaired if improper anesthetics are used, but also the recovery of PF and hemodynamics. In the present work, Sevo allowed patients in Group A to wake up more quickly than *P*, with better and effective recovery of PF and hemodynamics. In the study on the application of Sevo in elderly patients with lung cancer, Qin et al. [25] also suggested that compared with *P*, Sevo inhalation general anesthesia can more effectively improve PF with less effect on patients' cognitive function, which is consistent with our results.

In terms of postoperative complication rate and patient recovery, a lower complication rate and better recovery of various indicators were determined in Group A. It has been indicated that volatile anesthetics are safe and effective. The use of Sevo promotes early extubation and facilitates rapid transfer of patients from the operating room to the recovery room, which has a positive effect on patient recovery and restores the degree of respiratory protective reflexes and arousal as quickly as possible [26, 27]. *P* anesthesia is not only less effective than volatile anesthetics such as Sevo but also less safe, with greater side effects [28]. Therefore, the postoperative complication rate in Group A is lower, indicating better safety. In combination with these findings, Sevo has more favorable anesthetic effects, better recovery effects on PF and hemodynamics of patients, and higher safety than *P*, which explains better postoperative recovery in patients who used Sevo.

There are still many deficiencies in this study. Due to the limitations of research conditions, we were unable to detect the relevant molecular indicators of patients. Nor have we investigated patients' status during surgery and their satisfaction with the two surgical anesthesia methods. In future studies, we will supplement these tests while continuously improving the surgical procedures to facilitate patients' recovery.

## 5. Conclusion

Collectively, Sevo inhalation anesthesia has a better anesthetic effect for MO patients undergoing LBS, with a higher safety profile, which is worthy of clinical promotion [29].

## Figures and Tables

**Figure 1:** Time of recovery from anesthesia. (a) Eye-opening time: Group A presented shorter eye opening time than Group B (*P* < 0.05). (b) Intubation time: Group A had shorter intubation time than Group B (*P* < 0.05). (c) Directional force recovery time: the directional force recovery time was significantly shorter in Group A than in Group B (*P* < 0.05). Note: ^*∗*^*P* < 0.05 vs. Group B.

**Figure 2:** Hemodynamics. (a) Heart rate: After surgery, the heart rate of both groups showed significant changes, with a high level in Group A compared with Group B (*P* < 0.05). (b) Mean arterial pressure: There were significant changes in the mean arterial pressure in both groups after operation, and the level was significantly higher in Group A versus Group B (*P* < 0.05). Note: ^*∗*^*P* < 0.05 vs. Group B; ^#^*P* < 0.05 vs. after treatment.

**Figure 3:** Pulmonary function. (a) P_peak_: There were significant changes in P_peak_ in both groups postoperatively, with a lower _Ppeak_ in Group A versus Group B (*P* < 0.05). (b) Pplat: Postoperatively, the P_plat_ changed statistically in both groups and was lower in Group A (*P* < 0.05). Note: ^*∗*^*P* < 0.05 vs. Group B; ^#^*P* < 0.05 vs. after treatment.

**Figure 4:** Postoperative recovery. (a) Standard time out of PACU : The standard time out of PACU was significantly shorter in Group A than in Group B (*P* < 0.05). (b) Postoperative feeding time: Group A showed shorter postoperative feeding time than Group B (*P* < 0.05). (c) Hospital stay: The hospital stay was significantly shorter in Group A than in Group B (*P* < 0.05). Note: ^*∗*^*P* < 0.05 vs. B group.

**Table 1:** General data of two groups of patients.

Classification	Group A (*n* = 100)	Group B (*n* = 50)	*t*/*χ*^2^	*P*
Sex			0.487	0.485
Male	54 (54.00)	30 (60.00)		
Female	46 (46.00)	20 (40.00)		
Age (years)	47.10 ± 6.04	48.72 ± 6.43	1.080	0.284
BMI (kg/m^2^)	42.01 ± 3.08	42.70 ± 2.76	0.969	0.336

Family type			0.642	0.423
Nuclear family	83 (83.00)	44 (88.00)		
Others	17 (17.00)	6 (12.00)		

Place of residence			0.269	0.604
Urban	74 (74.00)	35 (70.00)		
Rural	26 (26.00)	15 (30.00)		

Drinking			0.085	0.770
Yes	80 (80.00)	41 (82.00)		
No	20 (20.00)	9 (18.00)		

Eating habits				
Heavy	75 (75.00)	36 (72.00)	0.156	0.693
Light	25 (25.00)	14 (28.00)		

**Table 2:** Incidence of complications after treatment in two groups.

	Group A (*n* = 100)	Group B (*n* = 50)	*χ* ^2^	*P*
Nausea	2 (2.00)	3 (6.00)	—	—
Vomiting	0 (0.00)	2 (4.00)	—	—
Labored breathing	0 (0.00)	1 (2.00)	—	—
Chills	1 (1.00)	4 (8.00)		
Complication rate	3 (3.00)	10 (20.00)	12.170	<0.001

## Data Availability

The labeled dataset used to support the findings of this study are available from the corresponding author upon request.
